The article "Effect of Foot Reflexology on Sexual Function of Patients under Hemodialysis: A Randomized Parallel Controlled Clinical Trial" was published in 2021. Journal: Evid Based Complement Alternat Med.

# Effect of Foot Reflexology on Sexual Function of Patients under Hemodialysis: A Randomized Parallel Controlled Clinical Trial

**DOI:** 10.1155/2021/8553549

**Published:** 2021-10-21

**Authors:** Somayeh Zeidabadinejad, Parvin Mangolian Shahrbabaki, Mahlagha Dehghan

**Affiliations:** ^1^Nursing Research Center, Kerman University of Medical Sciences, Kerman, Iran; ^2^Department of Critical Care Nursing, Razi Faculty of Nursing and Midwifery, Kerman University of Medical Sciences, Kerman, Iran

## Abstract

**Introduction:**

Hemodialysis patients experience sexual dysfunction due to the nature of their disease and its complications. Dialysis patients have reported sexual dysfunction as one of the most important stressors, which leads to many psychological and physiological problems. Sexual function in hemodialysis patients has been improved with pharmaceutical and nonpharmacological therapies. Foot reflexology is a complementary and alternative treatment that can be used in conjunction with contemporary care. By activating the chemical nerve system, reflexology may balance enzymes and regulate endocrine function.

**Objectives:**

To determine the effect of foot reflexology on the sexual function of hemodialysis patients.

**Methods:**

This randomized controlled trial was conducted on 47 patients on chronic hemodialysis referred to Imam Reza Hospital in Sirjan, Iran, who were divided into two groups of reflexology (*n* = 24; male = 19 and female = 5) and sham (*n* = 23; male = 18, and female = 5). The intervention group received foot reflexology during dialysis for four weeks, three times a week, 30 minutes each time (15 minutes per foot). The sham group received nonspecific foot massage without applying pressure on standard reflex points with the same condition and duration as the intervention group. The international index of erectile function and female sexual function index was assessed before, immediately, and one month after the intervention.

**Results:**

The results showed that immediately after the intervention, male orgasm function, sexual desire, and intercourse satisfaction in the reflexology group was significantly higher than those of the sham group. There was no significant difference between the two groups regarding erectile function and overall satisfaction. Furthermore, there was no significant difference between the two groups in terms of different aspects of female sexual function.

**Conclusions:**

Foot reflexology, as an effective intervention treatment, can reduce some aspects of sexual dysfunction of male patients under hemodialysis.

## 1. Introduction

Chronic kidney disease (CKD) is an irreversible kidney failure that has lasted for more than three months, and it is characterized by incurable and permanent loss of kidney function [1].

The article "Effect of Foot Reflexology on Sexual Function of Patients under Hemodialysis: A Randomized Parallel Controlled Clinical Trial" was published in 2021. Journal: Evid Based Complement Alternat Med.

The CKD mortality rate was 15.9% and 16.6% per hundred thousand people globally and in Iran in 2017, respectively [2]. It is predicted that 90,000 people in Iran will suffer from this disease by 2021 [3]. Kidney transplantation and dialysis, alternative therapies, are constant needs of patients with end-stage renal disease to survive [4]. According to available statistics, about 16% are added annually to patients undergoing hemodialysis in Iran [5].

The patients experience problems such as fatigue, decreased appetite, decreased sexual function, hypotension, muscle spasm, nausea and vomiting, headache, and pruritus due to kidney failure and related complications [6]. On the other hand, changes in the function of the hypothalamic-pituitary-gonadal axis (hormonal imbalance), neurovascular disorders, neuropsychological effects of the disease, and side effects of drugs can aggravate sexual dysfunction in such patients [7, 8]. Erectile dysfunction in men and orgasm dysfunction in women cause sexual dysfunction, so they cannot experience sexual satisfaction [9]. The prevalence of sexual dysfunction is 19% among patients with kidney failure and up to 70% in dialysis patients [10].

The severity of sexual dysfunction varies from one person to another, depends on the degree of kidney failure, and is often associated with decreased sexual pleasure. The severity of this disorder can vary from a slight decrease in sexual desire to failure to reach orgasm [8, 11]. While dialysis patients have reported sexual dysfunction as the most important stressor, sexual dissatisfaction can have consequences such as feelings of unhappiness and various psychological and physical consequences [6, 12]. It is important to design interventions that can reduce the complications of the disease and treatment in patients undergoing hemodialysis [13]. Pharmacological [14, 15] and nonpharmacological [7, 11] interventions have been used to improve sexual function of the patients undergoing hemodialysis [16].

Drug therapies have their own side effects, and healthcare systems prefer to use nonpharmacological therapies to treat patients. Today, complementary and alternative medicine, as a tolerable, complication-free therapy with minimal drug interaction has become more popular [17].

The World Health Organization (WHO) defined complementary and alternative medicine as indigenous knowledge, skills, beliefs, and experiences in different cultures that are used for health, prevention, recovery, or physical and mental therapy [18]. Complementary medicine is divided into biological therapies, including herbal medicines, vitamins, and dietary supplements, and nonbiological treatments such as acupuncture, hydrotherapy, massage, reflexology, and music therapy [19]. Reflexology, one type of complementary and alternative medicine, can be used as a nursing intervention along with modern medicine. The mechanism of action is that putting pressure to a specific area of the skin stimulates reflexes and transmits them to the brain, so reflexology balances enzymes and regulates endocrine function by stimulating the chemical nervous system [20].

The article "Effect of Foot Reflexology on Sexual Function of Patients under Hemodialysis: A Randomized Parallel Controlled Clinical Trial" was published in 2021. Journal: Evid Based Complement Alternat Med.

Reflexology balances and relaxes proactive areas and stimulates inactive areas of the body [21].

A systematic review of studies on sexual function showed contradictory results of aerobic exercises and no effect of resistance training on patients' sexual functions [22]. The effect of reflexology was studied on factors such as the severity of fatigue [23], depression [24], restless legs syndrome [25], pain, muscle cramps [26], sleep quality [27] of the hemodialysis patients, but no study has investigated the effect of reflexology on sexual function of the hemodialysis patients.

Concerning the nature of dialysis and its treatment conditions, it is necessary to identify and eliminate its complications, especially sexual dysfunction. On the other hand, the healthcare team may not pay attention to patients' sexual problems because patients were reluctant to express them due to the culture prevailing in the Iranian society. Therefore, the healthcare team should use different interventions such as different types of complementary medicine to reduce patients' problems. Reflexology, an easy, low-cost, and practicable method without complications, is a nursing intervention that can be used in combination with medical treatments during dialysis to reduce stress and balance the body by creating electrochemical messages and stimulating nervous points [28]. Since there was no sufficient evidence on the effect of reflexology on sexual function of the patients undergoing hemodialysis, the aim of this study was to investigate the effect of foot reflexology on sexual function of the patients undergoing hemodialysis.

## 2. Methods

### 2.1. Study Type and Setting

The present study is a randomized parallel controlled clinical trial performed on hemodialysis patients referred to Imam Reza Hospital in Sirjan, southeast of Iran, from August to October 2020.

### 2.2. Sample Size and Sampling

Concerning the limited study population, all patients undergoing hemodialysis in the study setting were purposefully evaluated. Out of 110 patients undergoing hemodialysis in the study setting, 55 patients met the inclusion criteria. Inclusion criteria were patients aged 18–65 years [29], who did not use drugs for sexual problems [29], were at least 3 months on hemodialysis [30] three times a week, four hours each time [25, 31], with no medical contraindications such as foot ulcers, amputation, and orthopedic problems [23, 32], no debilitating and chronic diseases such as cancer, chronic respiratory failure, heart failure, rheumatoid arthritis, Lupus erythematosus [17, 23], those who were married and living with a spouse [33–35], and with no known psychological problems such as depression and bipolar disorder according to the patient's self-declaration [29]. Exclusion criteria were medical contraindications (such as diabetic foot ulcers), death or divorce of a spouse, failure to perform the intervention in three consecutive sessions, and failure to complete the questionnaires.

The article "Effect of Foot Reflexology on Sexual Function of Patients under Hemodialysis: A Randomized Parallel Controlled Clinical Trial" was published in 2021. Journal: Evid Based Complement Alternat Med.

The third author allocated samples into two groups by stratified block randomization method (stratum: gender). Labels A or B (*A* = sham, *B* = foot reflexology) were assigned to the groups, and the block size was four. The randomization list was generated by using free online software (https://www.sealedenvelope.com/simple-randomiser/v1/lists). The third author generated the randomization list and the first author enrolled the participants and assigned them to the two groups. Power analysis calculations with G *∗* Power software (version 3.1.9.2) indicated that (power = 80%, *P*=0.05, number of groups = two, and number of measurements = three) 36 participants would be needed to detect an effect size of 0.4. Finally, eight subjects (four in the sham group and four in the reflexology group) were excluded from the study for various reasons (lack of cooperation, quadriplegia, diabetic foot, death, divorce) and the analysis was performed on 37 male samples and 10 female samples (Figure 1).

### 2.3. Data Collection Tool

Demographic and background information questionnaire, international index of erectile function (IIEF), and female sexual function index (FSFI) were used to achieve the research objectives.

Demographic and background information questionnaire includes gender, age, occupation, number of children, level of education, monthly income, duration of dialysis, duration of marriage, cause of kidney failure, physical activity, history of cardiovascular and diabetes diseases, history of smoking, history of other diseases, hypertension, history of taking hypertensive drugs, previous sexual problems, laboratory tests, serum factors such as hemoglobin, hematocrit, platelets, white and red blood cell count, serum albumin level, parathyroid hormone level, blood urea nitrogen, urea reduction ratio (URR), serum iron, ferritin, phosphorus, calcium, potassium, albumin, *K t/V* (dialysis adequacy = clearance multiplied by time/volume) and alkaline phosphatase.

The article "Effect of Foot Reflexology on Sexual Function of Patients under Hemodialysis: A Randomized Parallel Controlled Clinical Trial" was published in 2021. Journal: Evid Based Complement Alternat Med.

#### 2.3.1. The International Index of Erectile Function (IIEF)

The International Index of Erectile Function (IIEF) developed by Rosen et al. (1997) was used for the evaluation of male sexual function. The index is divided into five domains: erectile function (six items), orgasmic function (two items), sexual desire (two items), intercourse satisfaction (three items), and overall sexual satisfaction (two items). Items 1–9 are scored from zero to five, and items 10–15 are scored from one to five, with a higher score indicating more desirable sexual function [36]. Rosen reported its appropriate validity and reliability for the first time in 1997 (Cronbach's alpha: 0.82) [36]. With the opinion of experts, Pakpour et al. in Iran (2014) confirmed the content validity of the index. The index reliability was more than 70% by Cronbach's alpha method [37].

#### 2.3.2. The Female Sexual Function Index (FSFI)

The Female Sexual Function Index (FSFI) developed by Rosen et al. (1997) is a 19-item self-report inventory designed to assess female sexual function. It comprises six domains: desire (two items), subjective arousal (four items), lubrication (four items), orgasm (three items), satisfaction (three items), and pain (three items) [38]. The items 1–14 as well as 17–19 are scored from zero to five on a Likert scale and items 15 and 16 are scored from one to five. A score of zero indicates no sexual activity for at least 4 weeks. Since the number of items in each domain is not equal in FSFI, the scores obtained from the items of each domain are added together and multiplied by the factor number. The total score of the scale is obtained by sum of the scores of the six domains, with higher scores indicating better sexual function. The maximum score was six for each domain and 36 for the whole scale. The minimum score was 1.2 for sexual desire, 0 for arousal, lubrication, orgasm and pain, 0.8 for sexual satisfaction, and 2 for the whole scale. The cutoff points for the whole scale and subscales are 28, 3.3 (desire), 3.4 (subjective arousal), 3.4 (lubrication), 3.4 (orgasm), 3.8 (satisfaction), and 3.8 (pain). In other words, scores higher than the cutoff point suggests good function [38].

Rosen published its appropriate validity and reliability for the first time in 2000 (Cronbach's alpha: 0.89) [38]. Mohammadi et al. (2008) evaluated the validity and reliability of this index in two groups of women with sexual dysfunction and the control. The validity of the Persian version showed a significant difference between the mean scores of the whole scale and each of the domains in the case and control groups. Therefore, the results generally show acceptable and appropriate psychometric properties. The reliability of the scale and subscales was obtained by calculating the Cronbach's alpha coefficient, which was above 0.70 for the whole scale, indicating the good reliability [39].

The article "Effect of Foot Reflexology on Sexual Function of Patients under Hemodialysis: A Randomized Parallel Controlled Clinical Trial" was published in 2021. Journal: Evid Based Complement Alternat Med.

### 2.4. Intervention

The patient's privacy in the reflexology group was maintained before the intervention; the patient was placed in a quiet and bright room, and the researcher sat on a chair at the foot of the patient's bed and performed the massage. She first cleaned the patient's foot with cotton soaked in warm water, warmed her hands so as not to irritate the patient, and used one-two cc of baby oil to facilitate the massage. Before performing the main technique, she dedicated the first two minutes of each session to the relaxation technique, including back and forth movements of the palm on the outer edge of the foot from the outer ankle to the little toe to relieve muscle tension and spasm. Then, she took the heel of one foot in her left hand and applied alternating pressures on the relevant reflex points with her right thumb in a reciprocating manner [3, 40–42].

The reflex points in the present study were solar plexus, pituitary gland, kidney, pineal gland, heart, liver/spleen, adrenal, lung, stomach, ovary/testis, uterus/prostate [3, 35, 40–43]. She massaged and gently applied pressure on each of the above points for one minute based on the patient's tolerance [25].

At the end, she performed a general massage for two minutes. Thus, this protocol lasted 30 minutes (15 minutes per foot) for four weeks, three times a week. The researcher started the massage in the second hour of dialysis because the patient's condition was more balanced and the ward was less crowded due to routine care. Since the intervention took some time, the researcher could perform the exercise more peacefully and accurately. She learned reflexology under the supervision of a complementary medicine specialist and started the interventions and data collection after her approval.

Before the intervention, the patient in the sham group was placed in a quiet and bright room, and the researcher sat on a chair at the foot of the patient's bed and performed the massage. She first cleaned the patient's foot with cotton soaked in warm water, warmed her hands so as not to irritate the patient, and used one-two cc of baby oil to facilitate the massage. She massaged the foot without applying pressure on the standard reflex points with the same duration as the intervention group [24]. Thus, this protocol lasted 30 minutes (15 minutes per foot) for 4 weeks, 3 times a week. A researcher, who was unaware of the sample allocation, collected the data.

The article "Effect of Foot Reflexology on Sexual Function of Patients under Hemodialysis: A Randomized Parallel Controlled Clinical Trial" was published in 2021. Journal: Evid Based Complement Alternat Med.

Information about demographic characteristics, sexual function, and clinical information was obtained through interviewing both the intervention and sham groups. Data on sexual function were collected from both groups (intervention and sham), before, immediately, and one month after the intervention (follow-up).

### 2.5. Data Analysis

SPSS25 was used for data analysis. Frequency, percentage, mean, and standard deviation were used to describe the samples. Independent *t*-test and Mann–Whitney *U* test were used to compare the quantitative variable between the two groups. Chi-square test and Fisher's exact test were used to compare the qualitative variable between the two groups. Repeated-measures ANOVA test was used to compare the mean scores of different aspects of erectile function in men and sexual function in women, and Bonferroni post hoc test was used to evaluate comparisons within and between groups. Significance level was considered *p* < 0.05.

### 2.6. Ethical Considerations

The present study was done after obtaining the code of ethics no. IR.KMU.REC.1399.248 from the Ethics Committee of Kerman University of Medical Sciences and the code of clinical trial (IRCT20200712048085N1) from Iranian Registry of Clinical Trials, coordinating with the heads of Imam Reza Hospital in Sirjan and obtaining informed consent from eligible patients. After obtaining informed written consent from the patients, she explained them the objectives and method of the study before the intervention, and assured them about the information confidentiality and the safety of the study. At the end of the study, a procedure was invented to comply with the study's ethical principles, and interventions were granted to the sham group.

## 3. Results

### 3.1. Baseline Characteristics of the Participants

The mean ages of the samples in the foot reflexology group and sham group were 50.54 ± 2.38 and 50.43 ± 2.16, respectively (*p*=0.97). The two groups were homogenous in terms of spouse's age, duration of marriage, gender, level of education, number of children, occupation, monthly income, physical activity, spouse's level of education and occupation, history of addiction, and satisfaction with sexual function (*p* > 0.05) (Table 1).

No significant differences were found between the two groups in laboratory tests, KT/V and URR (*p* > 0.05) (Table 2).

### 3.2. Sexual Function in Men under Hemodialysis

According to Table 3, the mean scores of erectile function in the foot reflexology group were 12.0, 16.42, and 10.47 in *T*1, *T*2, and *T*3, respectively. The erectile function scores of men were significantly higher immediately after the foot reflexology than before and one-month after foot reflexology (*p* < 0.05). The erectile function scores of men in the sham group were 11.22, 11.28, and 9.0 in *T*1, *T*2, and *T*3, respectively. On the other hand, the erectile function scores decreased over time (*p* < 0.05). Although the erectile function scores of men in the foot reflexology group were higher than that of the sham group immediately after the intervention, it was not statistically significant; however, the effect size was 0.56.

The article "Effect of Foot Reflexology on Sexual Function of Patients under Hemodialysis: A Randomized Parallel Controlled Clinical Trial" was published in 2021. Journal: Evid Based Complement Alternat Med.

The orgasm function scores of men were significantly higher immediately after foot reflexology than before and one-month after foot reflexology (*p* < 0.05). The orgasm function scores of men in the sham group did not change over time (*p* > 0.05). The orgasm function scores of men in the foot reflexology group were significantly higher than that of the sham group immediately after the intervention (effect size = 0.76).

The sexual desire scores of men were significantly higher immediately after foot reflexology than before and one-month after foot reflexology (*p* < 0.05). The sexual desire scores of men in the sham group did not change significantly over time (*p* > 0.05). The sexual desire scores of men in the foot reflexology group were significantly higher than that of the sham group immediately after the intervention (effect size = 1.33).

The intercourse satisfaction scores of men were significantly higher immediately after foot reflexology than before and one-month after foot reflexology (*p* < 0.05). The intercourse satisfaction scores of men in the sham group did not change significantly over time (*p* > 0.05). The intercourse satisfaction scores of men in the foot reflexology group were significantly higher than that of the sham group immediately after the intervention (effect size = 0.67).

The overall satisfaction scores of men were significantly higher immediately after foot reflexology than before and one month after foot reflexology (*p* < 0.05). The overall satisfaction scores of men in the sham group did not change significantly over time (*p* > 0.05). Although the overall satisfaction scores of men in the foot reflexology group were higher than that of the sham group immediately after the intervention, it was not statistically significant; however, the effect size was 0.55.

### 3.3. Sexual Function in Women under Hemodialysis

According to Table 4, the total sexual function scores of women in the foot reflexology group were 11.58, 21.22, and 16.1 in *T*1, *T*2, and *T*3, respectively. On the other hand, the total sexual function scores of women were significantly higher immediately after foot reflexology than before and one-month after foot reflexology (*p* < 0.05). The total sexual function scores of men in the sham group were 19.88, 18.76, and 19.58 in *T*1, *T*2, and *T*3, respectively. The total sexual function scores of women in the sham group did not significantly change over time (*p* > 0.05). Although the total sexual function score of women in the foot reflexology group was higher than that of the sham group immediately after the intervention, it was not significantly different. The pattern of changes in the different sexual function domains in both groups was similar to the total score.

The article "Effect of Foot Reflexology on Sexual Function of Patients under Hemodialysis: A Randomized Parallel Controlled Clinical Trial" was published in 2021. Journal: Evid Based Complement Alternat Med.

### 3.4. Adverse Events

None of the participants in the foot reflexology group and the sham group reported any adverse effect.

## 4. Discussion

Hemodialysis patients suffer from sexual dysfunction greatly [9]. The results of the present study showed men's orgasm, sexual desire, and intercourse satisfaction significantly increased immediately after the intervention, but sexual function domains were not statistically significant in women, despite the increasing scores of all domains of sexual function immediately after the intervention. No study in the review of literature examined the effect of reflexology on sexual function of the hemodialysis patients. Therefore, studies similar to the present intervention were used.

Gozuyesil et al. reported the effectiveness of foot reflexology in improving the sexual function of women aged 40–60 years in Turkey [35]. However, Pedram Razi et al. showed that reflexology decreased sexual function and pleasure in women with breast cancer undergoing chemotherapy [43]. They used quality of life instrument in which sexual function was examined as one of the domains of quality of life.

Tirgari et al. demonstrated that the sexual rehabilitation program with sexual training and exercises related to pelvis could improve sexual function in men with coronary artery disease [44]. Gerbild et al. (2018) showed that moderately intense aerobic exercise, 40 minutes four times a week improved erectile function in men [45]. Stanton et al. (2018) reported the effectiveness of intense exercises in female sexual function [46]. Both sexes were examined simultaneously in the present study, but there is little evidence in this regard. Fergus et al. (2019) showed the effect of exercise on reducing erectile dysfunction in men and protecting women against sexual dysfunction [47]. Exercise seems to activate the sympathetic nervous system and endocrine stimulates sexual function in women physiologically [46]. The mentioned interventions with the mechanism of reflexology all have been effective in the nervous system, the balance of enzymes, regulation of the endocrine function, balance of the proactive areas, and stimulation of inactive areas of the body [20, 21].

The article "Effect of Foot Reflexology on Sexual Function of Patients under Hemodialysis: A Randomized Parallel Controlled Clinical Trial" was published in 2021. Journal: Evid Based Complement Alternat Med.

Exercise is also assumed to improve the arterial supply of the penis [47] and it is well known that the penis and clitoris are common in embryonic origin and both organs have erectile tissue, skeletal muscle, and nervous system [48]. On the other hand, reflexologists believe that the foot is a reduced map of the whole body and reflects all the organs and parts of the body, and the arrangement of the body parts on the foot corresponds to their orders in the body [49]. Massage of these points using unique techniques increases blood flow to the related organs and helps repair damaged areas [50]. The results of Doppler ultrasound in a study showed that reflexology of the kidney area in the soles increased the blood flow to the kidneys compared with the group that did not receive reflexology [51]. Both exercise and reflexology may improve sexual activities by increasing the blood flow to sexual organs.

Carcelén-Fraile et al. (2020) showed that resistance training, unlike aerobic exercise, did not affect female sexual function and quality of sexual life [22]. It is noteworthy that in previous studies, intervention was done more on the pelvic muscles [22, 44] and less on the feet.

The mechanism of acupressure is similar to that of reflexology based on meridians, energy highways of the body [52]. Wang et al. (2014) in China showed an increase in sexual function of the auricular acupressure group 3, 6, and 9 months after the start of the intervention compared with the control group [53].

Studies have been conducted on acupuncture and contradictory results have been reported. Cui et al. (2016) and Li et al. (2017) showed that the therapeutic effect of acupuncture on erectile dysfunction was controversial [54, 55]. Meanwhile, Bay et al. (2019) reported the positive effect of acupuncture on male sexual function [56], but its safety and complications have not been adequately studied [54]. Foot reflexology can be used to improve the sexual function of hemodialysis patients because it is safe, with no complications and requires no special equipment compared with acupuncture.

In the present study, the effect of reflexology on changes in male sexual desire was significant, but changes in female sexual desire were not significant, despite the increasing scores of all domains of sexual function immediately after the intervention. The reason is insufficient number of female samples in both massage and sham groups (five samples in each group). Among the strengths of massage performed in this study were the massage duration (15 minutes for each foot in 12 sessions) and massage of 12 points on the foot. Even the points related to the sexual organs on the foot, including the uterus/prostate and ovaries/testicles, were massaged, but in the study of Razi et al. (2013), not all of these points were massaged [43].

The article "Effect of Foot Reflexology on Sexual Function of Patients under Hemodialysis: A Randomized Parallel Controlled Clinical Trial" was published in 2021. Journal: Evid Based Complement Alternat Med.

Organic and metabolic disorders and physiological changes associated with chronic kidney failure in hemodialysis patients cause them to experience psychological symptoms that disrupt their lifestyle and create sexual problems [57, 58]. Addressing sexual function in hemodialysis patients is important because although many of the symptoms of kidney failure are resolved with dialysis, sexual dysfunction persists throughout the treatment course and hemodialysis patients are less interested in sex [59]. Therefore, it is more difficult to manage the problems of such patients. Reflexology, a type of complementary and alternative medicine, has a long history and is used in combination with modern medicine as a holistic approach, a nursing intervention, and a discipline that supports traditional care [60].

Diseases are caused by energy blockage in the body, and stimulation of reflex points may eliminate these blockages and release energy in the body [61]. Evidence shows strong physiological and psychological effects of foot reflexology and no destructive effects have been reported in specific medical conditions [62]. According to the available evidence and the results of the present study, health care providers can use this intervention to improve sexual function of the patients undergoing hemodialysis.

This study has several limitations. Some of the hemodialysis patients were reluctant to complete the study questionnaires because of the chronic disease process, so we asked them to complete the questionnaires when they were in a good condition. As the level of pressure to the feet depended on the patient's tolerance, it was adjusted with the patient's tolerance. To reduce possible errors during the intervention, the researcher was trained by a complementary medicine specialist and performed the interventions after her approval. Low sample size, particularly in the case of females, was another limitation of the study. More studies with larger sample size are needed to confirm the present study results. Furthermore, we did not use Penile Doppler Ultrasonography for assessing the severity of vascular impotence. Different severity of vascular impotence could affect the study results. In addition, the psychological status of patients plays an essential role in sexuality. Although we considered the psychological disorders as noninclusion criterion, the psychological status of participants during the study may have had an impact on their sexual function.

The article "Effect of Foot Reflexology on Sexual Function of Patients under Hemodialysis: A Randomized Parallel Controlled Clinical Trial" was published in 2021. Journal: Evid Based Complement Alternat Med.

## 5. Conclusion

The results of the present study showed the significant effect of foot reflexology on men's orgasm, sexual desire, and intercourse satisfaction. Since sexual dysfunction is one of the most common problems in these patients, reflexology as an effective, simple, low-cost, and practical intervention can reduce some sexual problems of such patients due to their special conditions and limitations in drug use. Therefore, nurses in hemodialysis centers can learn reflexology and provide it to patients. Due to the limited evidence on the domains of sexual function in men and women, further studies are needed to confirm the effects of foot reflexology on sexual function, especially in women, and it is suggested that future studies be conducted on larger samples in different hemodialysis centers.

## Figures and Tables

**Figure 1:** The study flow diagram.

**Table 1:** Comparison of demographic and clinical information in patients of reflexology and sham groups.

Variable	Group					
	Reflexology (*n* = 24)		Sham (*n* = 23)		Statistical test	*p* value
	Mean	SD	Mean	SD		
Age	50.54	2.38	50.43	2.16	*T* = −0.03	0.97
Spouse's age	47.58	2.76	45.09	1.97	*Z* = −0.31	0.76
Duration of marriage	24.29	3.13	25.26	2.25	*Z* = −0.50	0.62
	Frequency	Percent	Frequency	Percent	Statistical test ^*∗*^	*p* value
Sex					0.006	0.94
Female	5	20.8	5	21.7		
Male	19	79.2	18	78.3		

Education level					1.73	0.19
Middle/high school	17	70.8	12	52.2		
Diploma/higher	7	29.2	11	47.8		

No. of children					4.09	0.39
None	5	20.8	2	8.7		
1	2	8.3	3	13		
2	5	20.8	7	30.4		
3	5	20.8	8	34.8		
>4	7	29.2	3	13		

Job					0.62	0.73
Unemployed/housewife	13	54.2	10	43.5		
Employed	7	29.2	9	39.1		
Retired	4	16.7	4	17.4		

Monthly income					1.84	0.40
<1000000 tomans	16	66.7	12	52.2		
1000000–2000000 tomans	6	25	6	26.1		
>2000000 tomans	2	8.3	5	21.7		

Physical activity					2.51	0.32
None	15	62.5	14	60.9		
Sometimes	8	33.3	5	21.7		
Regularly	1	4.2	4	17.4		

Spouse's education					1.04	0.31
Middle/high school	14	58.3	10	43.5		
Diploma/higher	10	41.7	13	56.5		

Spouse's job					4.14^*∗*^	0.16
Unemployed/housewife	16	66.7	17	73.9		
Employed	4	16.7	6	26.1		
Retired	4	16.7	0	0		

Spouse's smoking					0.27^*∗*^	0.67
Yes	2	8.3	3	13		
No	22	91.7	20	87		

Marital satisfaction before kidney failure					1.43^*∗*^	0.60
Poor	2	8.3	1	4.3		
Moderate	3	13.5	1	4.3		
Good	19	79.2	21	91.3		
Spouse's marital satisfaction before kidney failure					2.16^*∗*^	0.42
Poor	0	0	1	4.3		
Moderate	5	20.8	2	8.7		
Good	19	79.2	20	87		

*t* = independent *t*-test, *Z* = Mann–Whitney *U* test,  ^*∗*^Fisher's exact test, and chi-square test in other cases.

The article "Effect of Foot Reflexology on Sexual Function of Patients under Hemodialysis: A Randomized Parallel Controlled Clinical Trial" was published in 2021. Journal: Evid Based Complement Alternat Med.

**Table 2:** Comparison of laboratory tests of patients under hemodialysis between the two groups of foot reflexology and sham.

Variable	Group					
	Foot reflexology (*n* = 24)		Sham (*n* = 23)		Independent *t*-test	*p* value
	Mean	SD	Mean	SD		
KT/V	1.44	0.05	1.44	0.08	−0.03	0.98
Urea reduction ratio	0.68	0.01	0.68	0.02	−0.41	0.69
Albumin (g/dl)	3.63	0.07	3.82	0.1	1.60	0.12
Blood urea nitrogen (mg/dl)	106.71	4.85	112.04	6.15	0.68	0.50
Creatinine (mg/dl)	6.94	0.45	6.95	0.36	0.02	0.99
Fasting blood sugar (mg/dl)	99.42	13.39	108.43	11.45	0.51	0.61
Potassium (mEq/L)	5.13	0.18	5.05	0.15	−0.34	0.73
Sodium (mEq/L)	139.58	1.02	138.60	0.57	−0.83	0.41
Calcium (mg/dl)	9.13	0.18	8.99	0.20	−0.54	0.59
Phosphor (mg/dl)	5.43	0.22	5.40	0.28	−0.08	0.94
White blood cell (1000/mm^3^)	6.79	0.43	6.51	0.36	−0.50	0.62
Red blood cell (1,000,000/mm^3^)	4.28	0.13	4.17	0.11	−0.62	0.54
Hematocrit (%)	37.26	1.58	36.20	1.67	−0.46	0.64
Hemoglobin (g/dl)	11.83	0.44	11.68	0.28	−0.28	0.78
Platelet (1000/mm^3^)	153.17	8.48	155.04	9.13	0.15	0.88
Iron (mcg/dl)	497.26	259.56	332.67	271.17	−1.89	0.07
Ferritin(mg/dl)	287.50	263.99	270.68	247.95	0.68	0.50
Parathyroid hormone (ng/ml)	240.45	206.12	287.50	264.0	0.61	0.55
Alkaline phosphatase (IU/L)	263.68	143.28	266.56	144.57	0.06	0.95

SD: standard deviation; IU: international unit.

**Table 3:** Comparison of male sexual function and its domains between the two groups of foot reflexology and sham.

Male sexual function		Group									
		Foot reflexology (*n* = 19)			Sham (*n* = 18)			Mean difference		*p* value^*∗*^	Effect size
		Median	Mean	SD	Median	Mean	SD	Mean	SE		
Erectile function	*T*1	14	12.0	9.94	6.0	11.22	9.21	0.78	3.15	0.81	0.08
	*T*2	14	16.42	9.33	7.0	11.28	9.05	5.14	3.02	0.10	0.56
	*T*3	11	10.47	8.27	1.0	9.0	10.36	1.47	3.07	0.64	0.16

Orgasmic function	*T*1	4.0	3.74	3.38	2.0	4.0	3.16	−0.26	1.08	0.81	0.07
	*T*2	6.0	5.95	2.55	2.5	3.72	3.30	2.22	0.97	0.03	0.76
	*T*3	4.0	3.47	2.93	0.0	2.78	3.57	0.70	1.07	0.52	0.21

Sexual desire	*T*1	4.0	4.21	1.93	4.0	4.06	2.07	0.16	0.66	0.82	0.07
	*T*2	6.0	6.0	1.29	3.5	3.83	1.92	2.17	0.54	<0.001	1.33
	*T*3	4.0	3.68	1.83	2.0	3.39	1.88	0.29	0.61	0.63	0.16

Intercourse satisfaction	*T*	6.0	5.0	4.31	3.5	4.94	4.05	0.06	1.38	0.97	0.01
	*T*2	7.0	7.21	3.55	4.5	4.72	3.86	2.49	1.22	0.049	0.67
	*T*3	5.0	4.53	3.64	0.0	3.44	4.34	1.08	1.32	0.42	0.27

Overall satisfaction	*T*1	3.0	3.95	2.34	2.5	3.89	2.47	0.06	0.79	0.94	0.02
	*T*2	4.0	5.37	2.81	2.5	3.94	2.36	1.42	0.86	0.10	0.55
	*T*3	2.0	3.58	1.98	2.0	3.83	2.68	−0.25	0.77	0.74	0.11

^*∗*^Repeated-measures analysis of variance: adjustment for multiple comparisons: Bonferroni. T1: before intervention, T2: immediately after intervention, T3: one month after intervention, SD: standard deviation, and SE: standard error.

The article "Effect of Foot Reflexology on Sexual Function of Patients under Hemodialysis: A Randomized Parallel Controlled Clinical Trial" was published in 2021. Journal: Evid Based Complement Alternat Med.

**Table 4:** Comparison of female sexual function and its domains between the two groups of foot reflexology and sham.

Female sexual function		Group									
		Foot reflexology (*n* = 5)			Sham (*n* = 5)			Mean difference		*p* value^*∗*^	Effect size
		Median	Mean	SD	Median	Mean	SD	Mean	SE		
Desire	*T*1	1.8	2.16	1.24	2.4	2.76	1.17	−0.60	0.76	0.46	0.50
	*T*2	2.4	3.36	1.56	3.0	2.52	0.98	0.84	0.83	0.34	0.64
	*T*3	1.8	2.40	1.75	3.6	2.88	1.30	−0.48	0.98	0.64	0.31

Arousal	*T*1	1.8	2.22	1.87	2.7	3.18	2.32	−0.96	1.33	0.49	0.46
	*T*2	3.3	3.48	1.46	2.7	2.82	1.97	0.66	1.01	0.56	0.38
	*T*3	2.7	2.76	1.33	3.3	3.24	2.41	−0.48	1.23	0.71	0.22

Lubrication	*T*1	1.2	1.68	2.17	1.8	2.58	2.18	−0.9	1.38	0.53	0.41
	*T*2	2.4	2.94	1.48	2.4	2.7	1.9	0.24	1.08	0.83	0.14
	*T*3	2.1	2.46	1.22	1.8	2.58	2.15	−0.12	1.11	0.92	0.07

Orgasm	*T*1	1.2	1.2	1.47	4.0	2.8	2.08	−1.6	1.14	0.20	0.89
	*T*2	2.8	2.72	1.56	2.8	2.48	1.73	0.24	1.04	0.82	0.14
	*T*3	2.4	2.16	1.25	3.6	2.88	2.03	−0.72	1.07	0.52	0.43

Satisfaction	*T*1	1.2	1.60	1.36	4.0	3.6	1.67	−2.0	0.96	0.07	1.31
	*T*2	2.4	3.36	1.80	3.6	3.68	1.80	−0.32	1.14	0.79	0.18
	*T*3	2.4	2.48	1.28	3.6	3.44	1.89	−0.96	1.02	0.37	0.59

Pain	*T*1	2.4	2.72	2.82	6.0	4.96	1.73	−2.24	1.48	0.17	0.96
	*T*2	6.0	5.36	1.04	6.0	4.56	2.60	0.80	1.25	0.54	0.40
	*T*3	4.8	3.84	2.60	6.0	4.56	2.60	−0.72	1.64	0.67	0.28

Total	*T*1	11.4	11.58	10.07	19.3	19.88	10.48	−8.3	6.5	0.24	0.81
	*T*2	17.7	21.22	7.36	19.3	18.76	10.56	2.46	5.76	0.68	0.27
	*T*3	13.8	16.10	7.67	21.3	19.58	11.62	−3.48	6.22	0.59	0.35

^*∗*^Repeated-measures analysis of variance: adjustment for multiple comparisons: Bonferroni. T1: before intervention, T2: immediately after intervention, T3: one month after intervention, SD: standard deviation, and SE: standard error.

## Data Availability

Data will be made available by contacting with the corresponding author by e-mail.
